# microRNA-128 mediates CB1 expression and regulates NF-KB/p-JNK axis to influence the occurrence of diabetic bladder disease

**DOI:** 10.1186/s12967-020-02406-9

**Published:** 2020-07-16

**Authors:** Xin Gou, Jing Wu, Mingqing Huang, Yuting Weng, Tongxin Yang, Tao Chen, Guiqing Li, Kewei Fang

**Affiliations:** 1 Department of Urology, The Second Affiliated Hospital of Kunming Medical University, No. 374, Dianmian Dadao, Kunming, Yunnan 650101 People’s Republic of China; 2 Department of Biochemistry and Molecular Biology, The Primary Medicine School of Kunming Medical University, Kunming, 650101 People’s Republic of China; 3 Department of Urology, The 2nd Hospital of Kunming Medical University, Kunming, 650101 People’s Republic of China

**Keywords:** microRNA-128, CB1, Diabetes, Bladder disease, NF-KB, P-JNK, Apoptosis

## Abstract

**Background:**

Diabetic bladder disease is common complications of diabetes, its symptoms are diverse, can be due to different stages. In this study we investigate the mechanism of miR-128 targeting CB1 expression to mediate the occurrence of diabetic bladder disease.

**Methods:**

Bioinformatics analysis predicts related regulatory factors of miR-128 in diabetic bladder disease. Models of diabetic bladder lesions were constructed in male SD rats by intraperitoneal injection of streptozotocin at 65 mg/kg body weight. The expression of miR-128 and CB1 mRNA in bladder tissues of each group was detected by RT-qPCR, and CB1, NF-KB, p-JNK and Bcl2 protein expression was detected by Western Blotting. We tested the function of the bladder by urodynamics, detected the pathological characteristics of the bladder tissue by HE staining, and verified the targeting relationship between miR-128 and CB1 through the prediction of the biological website, dual luciferase reporter gene assay and RIP.

**Results:**

miR-128 was highly expressed in the bladder tissue of diabetic rats. Inhibition of miR-128 could improve the occurrence of diabetic bladder lesions in rats. miR-128 could target the inhibition of CB1 expression, and high expression of CB1 could antagonize miR-128 against diabetic bladder. In the diabetic bladder, miR-128 can regulate the expression of NF-KB and p-JNK through CB1 and affect the level of apoptosis. miR-128 regulates NF-KB/p-JNK through CB1, thus affecting the occurrence of diabetic bladder disease.

**Conclusion:**

The high expression of miR-128 can down-regulate the expression of CB1, promote the activation of NF-KB and p-JNK, increase the level of apoptosis and promote the occurrence of diabetic bladder disease.

## Background

Diabetic bladder disease is common complications of diabetes, its symptoms are diverse, can be due to different stages, but mainly manifested by impaired feeling of bladder filling and weakened contractility changes in urination characteristics, and may be complicated by urinary tract infection and bladder urination Tube reflux, hydronephrosis, kidney stones, and eventually uremia [1]. The number of people with diabetes has continued to increase in recent years [2]. Diabetic cystitis (DCP) is a systemic disease associated with diabetes in the urinary system of humans and animals, accounting for more than 80% of people with diabetes [3]. The pathogenesis of DCP is still unclear, it is a complex and has many incentives, and the course of the disease is closely related to time. Myogenic, currently considered neurogenic and urethral epithelial changes are the main causes of DCP [4, 5]. Many studies have tried to elucidate the mechanism of DCP, but it is still unclear. Therefore, the treatment of DCP is greatly restricted [6].

miRNAs are a group of highly conserved small RNA molecules that can regulate gene expression functions More and more studies show that miRNAs play an important role in many physiological processes [7, 8]. Mutations or disorders of miRNAs are related to a variety of human tumors. Over control protein coding to play a role in promoting or suppressing cancer [9]. Studies have shown that miR-128 expression in tumors of the nervous system, breast and prostate cancer, tumor expression is down-regulated [10], and through its target genes such as the oncogene Bmi-1 [11], EGFR [12], p70S6K1 [13], E2F3 [14], miR-128 play a role in suppressing cancer. However, level of miR-128a and its downstream regulated signals in diabetes have not been reported.

Recent years more reports were focused on the role of miR-144, also like miR-128 carcinogenesis because it is dysregulated and involved in the tumorigenesis of various cancer, such as lung cancer [15], osteosarcoma [16], hepatocellular carcinoma [17], thyroid cancer [18], bladder cancer [19] and colorectal carcinoma [20]. However, the biological functions and underlying molecular mechanism of miR-144 in DCP are not yet described. Therefore, we investigate the biological role and potential mechanism of miR-144 in DCP by several experiments in vitro and tumor growth of xenograft in vivo and in vitro.

## Methods

### Bioinformatics analysis

Through bioinformatics website microT (http://diana.imis.athena-innovation.gr/DianaTools/index.php?r=microT_CDS/), TargetScan (http://www.targetscan.org/vert_72/), miRWalk (http://mirwalk.umm.uni-heidelberg.de/) and RNAInter (http://www.rna-society.org/rnainter/), the downstream target genes of miR-128 in rats were jointly predicted using different binding site matching algorithms. We used the jvenn tool (http://jvenn.toulouse.inra.fr/app/example.html) to take the intersection of four predicted results for target gene screening. The interaction between genes was analyzed through the STRING website (https://string-db.org/), and the results of the interaction analysis were visualized using Cytoscape 3.5.1. In order to further predict the downstream regulatory factors of genes, we set the keyword “diabetic bladder disease” through the GeneCards database (https://www.genecards.org/) to find related genes, and used the STRING website to analyze the gene interactions. The relationship predicted downstream regulatory genes. The co-expression relationship of downstream genes was obtained through Chipbase v2.0 website (http://rna.sysu.edu.cn/chipbase/).

### Establishment of Diabetic Mellitus (DM) rat model

A total of 100 SPF male SD rats (purchased from the Experimental Animal Center of China Medical University), weighing 180–250 g, were randomly divided into 3 groups after fasting for 12 h: normal control group (NC group, n = 16); Polyuria control group (PU group, n = 16), hypertonic polyuria induced with 5% sucrose water as drinking water; diabetes group (DM group, n = 68), single intraperitoneal injection of streptozotocin (STZ; dissolved at pH = 4.2 in 0.1 mol/L framic acid buffer; Sigma, St. Louis, MO) at 65 mg/kg body weight. The rats in the NC group and the PU group were intraperitoneally injected with the same dose of normal saline. At 4 weeks after STZ injection, the blood glucose level was confirmed to be above 300 mg/dl, and the rats with urine glucose test strip ++++ were diabetic rats. All rats were free to eat and drink. At 6 and 12 weeks, 8 rats were randomly selected from each group, placed in a metabolic cage, and urine of rats was collected and weighed for 24 h, and then performed with urodynamic experiments. This experimental procedure and animal use protocol have been approved by the Animal Ethics Committee of the Second Affiliated Hospital of Kunming Medical University.

### Grouping and processing of experimental animals

The rats in the NC group, the PU group, and the successfully modeled DM group were anaesthetized with 200 g/L urethane (injection dose 1.5 g/kg) after 6 h of fasting. Ureter is inserted through the urethra to empty the urine after anesthesia. The rats in the NC group and the PU group were perfused with 0.2 ml of PBS solution through the ureter. There were 56 of DM group successfully modeled rats, and the modeling success rate was 93.33%. The modeled rats were divided into the following groups, 8 in each group: mimic NC group (urinary catheter perfusion with 0.2 mL mimic NC), miR-128 mimic group (urinary catheter perfusion with 0.2 mL miR-128 mimic), inhibitor NC group (urinary catheter perfusion with 0.2 mL inhibitor NC), miR-128 inhibitor group (urinary catheter perfusion with0.2 mL miR-128 inhibitor), mimic NC + oe-NC group (urinary catheter perfusion with mimic NC and oe-NC lentivirus 0.2 mL), miR-128 mimic + oe-NC group (urinary catheter perfusion with miR-128 mimic and oe-NC lentivirus 0.2 mL), and miR-128 mimic + oe-CB1 group (urinary catheter perfusion with miR-128 mimic and oe-CB1 0.2 mL each). miR-128 mimic/inhibitor, oe-CB1 and nonsense NCs were purchased from Shanghai GenePharma Co., Ltd. (Shanghai, China) packaged with lentivirus, and the virus injection volume was 2 × 10^7^ TU (Shanghai Gima Pharmaceutical Technology Co., Ltd.). The ureter was ligated after perfusion, and the bladder perfusate was retained for 2 h. At 12 weeks after STZ injection, rats in each group were examined for urodynamics. All rats had free access to water and were fed on a standard diet. This experimental procedure and animal use protocol have been approved by the Animal Ethics Committee.

### Urodynamic examination

Urotan (1200 mg/kg body weight) was used for urodynamic examination under subcutaneous anesthesia. The midline incision was taken to expose the bladder, and a 27-gauge trocar was used to puncture the catheter through the top of the bladder. The intravesical catheter was connected to a baroreceptor (-Nihon Kohden, Japan) and a microperfusion pump (-JMS, Japan) through a three-way valve. The bilateral ureters were severed near the entrance to the bladder and the distal ends were ligated. Use up your bladder. After 30 min of stabilization, 37 °C physiological saline was infused into the bladder at a rate of 0.08 ml/min, and a complete bladder manometry was performed. Record the bladder volume (the volume of physiological saline perfused until urination), the volume of single urination (the volume of physiological saline discharged through the urethral orifice), the maximum pressure in the bladder (the peak pressure in the bladder during urination), bladder compliance and disability urine volume (the amount of remaining normal saline aspirated through an intravesical catheter after urination). Calculate urination rate = urination volume × 100%/bladder volume. The above indicators are the average of 3 experiments.

### Bladder specimen processing and HE staining

After urodynamic examination, rats were euthanized by 3% pentobarbital sodium (P3761, Sigma, USA) anesthesia, the bladder was removed, the surrounding fat and connective tissue were removed, used paper to dry the bladder, and the bladder, was weighed. The complete bladder specimen was cut into the longitudinal muscle bundle of the bladder sidewall in Krebs buffer. The muscle bundle specimens were sectioned about 1 mm into 4% paraformaldehyde overnight, washed 3 times in PBS, shaked vigorously to wash the residual paraformaldehyde, and soaked in 70% alcohol solution overnight. After soaked in 80% and 90% alcohol solution for 1 h, sections were immerse 3 times in 100% alcohol for 1 h each time; xylene transparent 2 times for 8 min each time; immerse the wax in the oven at 65 °C (pre-melted) for 3 h, embed in paraffin, and use Leica LM2300 Type paraffin microtome, cut into 5 μm thick cross sections.

Sections were routinely dewaxed (3 times with xylene, 5 min/time) and hydrated (3 times with 100% alcohol, 90%, 80%, 70% alcohol once, 5 min/time), rinsed under running water. After 10 min of nucleus staining by hematoxylin, the excess hematoxylin stain was washed away with tap water. And then the sections were separated by 1% hydrochloric acid alcohol for 5 s, returned to blue by 1% ammonia for 5 s, and then the sections were washed with running water for 5 min. After Eosin staining for 3 min, the sections were treated with 80% ethanol and 90% ethanol for 5 s each, 100% ethanol 3 times for 5 min each, xylene transparent treatment 3 times for 5 min each, neutral gum seals, and then placed in a fume hood at room temperature and observed by Microscopy.

### RT-qPCR

About 30 mg of bladder tissue was excised, and total RNA was extracted by Trizol (15596026, Invitrogen, Car, Cal, USA) method. RNA was reverse transcribed into cDNA according to the instructions of the PrimeScript RT reagent Kit (TaKaRa Bio, Japan) reverse transcription kit. Primers were designed and synthesized by Shanghai Sangon Biotech (Table 1). The reaction solution was taken for real-time quantitative PCR operation. The reaction system was 20 μl: 10 μl SYBR Premix, 2 μl of cDNA template, 0.6 μl each of upstream and downstream primers, and 6.8 μl of DEPC water. RT-qPCR experiments were performed using a 7500-type fluorescent quantitative PCR from American Applied Biosystems company. 2^−∆∆Ct^ represented the doubling relationship of the target gene expression between the experimental group and the control group, the formula was as follows: ∆Ct = CT (target gene)-CT (internal reference), ∆∆Ct = ∆Ct experimental group-∆Ct control group. Ct is the number of diffusion cycles that the real-time fluorescence intensity of the reaction reaches when the threshold is set. At this time, the diffusion increases in a logarithmic phase. The expression of miR-128 and CB1 in the cells was calculated.

**Table 1:** Primer sequences used for RT-qPCR

Targets	Forward primer (5′–3′)	Reverse primer (5′–3′)
miR-128	CAGATCGTCACAGTGAACC	\
CB1	CGTCTGAGGATGGGAAGGTA	TCTTGACCGTGCTCTTGATG
GADPH	CTTCACCACCATGGAGAAGGC	GGCATGGACTGTGGTCATGAG

### Western blotting

About 100 mg of bladder tissue were lysed by RIPA lysate with a final concentration of 1 mM phenylmethylsulfonyl fluoride (PMSF). Protein quantification was performed using the Bio-Rad DC Protein Assay Kit (Guangzhou Yuwei Biotechnology Instrument Co., Ltd., Guangzhou, China). Each sample was added SDS loading buffer. And boiling in water for 10 min, the sample was load on a 10% SDS–polyacrylamide gel and run at 120 V, 30 min, and 100 V for 90 min. The protein was transferred from the gel to a PVDF membrane. The membrane was immersed in 1 × TBST containing 5% skimmed milk powder and gently shaken at room temperature for 2 h to block non-specific binding sites. PVDF membrane was wash 1 × TBST 3 times, 5 min/time. Add primary antibodies (anti-CB1, rabbit, 1: 250; Anti-NF-kB p65, rabbit, 1: 1000; anti-p-JNK, rabbit, 1: 1000; Abcam), incubated at 4 °C overnight, washed 3 times with 1 × TBST, 5 min/time, and then added with secondary antibody IgG (Affinity Biosciences Bio, S0001, goat anti-rabbit, 1: 20000) respectively and incubated 3 times with 1 × TBST at room temperature for 1 h. Development was performed with ECL. The gray value of Western blotting experimental protein expression was determined by Image J software, and the experiment was repeated three times.

### Dual luciferase report detection

The biological prediction website was used to analyze the binding site of miR-128 and CB1, and obtain the fragment sequence containing the action site. The 3′UTR region of CB1 was cloned and amplified into pmirGLO (E1330, Promega Corporation, USA), Luciferase vector named pWt-CB1. pMut-CB1 vector was constructed, pRL-TK vector (E2241, Promega Corporation, USA) expressing Renilla luciferase was constructed, and mimic NC and miR-128 mimic, sh-NC and sh-CB1 were co-transfected with reporter vector (CRL-1415, ATCC, USA) into bladder epithelial cells SV-HUC-1. Dual Luciferase Reporter Gene Assay Kit (GM-040502A, Qcbio Science&Technologies Co., Ltd., China) was used to measure the fluorescence intensity at 560 nm (Firefly RLU) and 465 nm (Renal RLU), and the ratio of firefly RLU/renal RLU was used to determine the binding intensity.

### RIP

In the experiment, the binding of miR-128, CB1 and Ago2 protein was detected according to the Magna RIP RNA-Binding Protein Immunoprecipitation Kit (Merck Millipore, USA). Lyse the cells with RIPA lysate for 5 min in an ice bath, and centrifugated at 4 °C for 10 min to remove the supernatant. Part of the cell extract was taken as input, and part was incubated with antibodies for co-precipitation. The specific steps were as follows: each co-precipitation reaction system was washed with 50 μL magnetic beads, resuspended in 100 μL RIP Wash Buffer, and 5 µg of antibody was added according to the experimental grouping. The magnetic bead-antibody complex was washed and resuspended in 900 μL RIP Wash Buffer, and 100 μL of cell extract was added and incubated overnight at 4 °C. The sample was placed on a magnetic holder to collect the magnetic bead-protein complex. Samples and Input were digested with proteinase K to extract RNA for subsequent PCR detection. Ago2 was mixed at room temperature for 30 min, and IgG was used as a negative control.

### Statistical analysis

SPSS 21.0 (IBM Corp., Armonk, NY, USA) was used for statistical analysis. The measurement data were expressed by mean ± standard deviation, and the two sets of data were compared using an unpaired design with normal distribution and uniform variance, and an unpaired t test was used. Data comparison among multiple groups was performed using one-way analysis of variance (ANOVA) and Tukey’s post hoc test. Data comparison between groups at different time points was performed using repeated measures ANOVA and post hoc testing was performed using Bonferroni. The relationship between the two indicators was analyzed using Pearson correlation. The difference was statistically significant at P < 0.05.

## Results

### miR-128 is highly expressed in bladder tissues of DM modeled rats

At 6 W and 12 W after STZ injection, 8 rats were randomly selected from each group for physiological characteristics observation. Compared with the NC group, the average blood glucose level of the rats in the DM group was significantly increased (P < 0.05), while the blood glucose level of the rats in the PU group was not significantly changed (Fig. 1a), and that of the rats in the DM group was significantly higher than that of the PU group (P < 0.05). Compared with the initial weight of the rats, the body weight of rats in the DM group was significantly lower than that of the NC group and the PU group during the same period (P < 0.05), while there was no significant difference in rat weight (Fig. 1b). Urine was collected through a metabolic cage. The results showed that compared with the NC group, the daily urine output of the rats in the PU group and the DM group was significantly increased (P < 0.05), and there was no significant difference between the PU group and the DM group (Fig. 1c) At the same time, there was no significant difference in the 24-h mean urine volume between 6 W and 12 W after STZ injection. After urodynamic examination, the bladder of each group was removed and weighed. As a result, compared with the NC group, the average weight of the bladder of rats in the PU group and the DM group increased significantly (P < 0.05). There was no difference between the PU group and the DM group, so was those at 6 W and 12 W after STZ injection (Fig. 1d).

**Fig. 1:** Identification of a diabetic bladder disease model in rats. **a** Statistical chart of blood glucose levels in rats; **b** Statistical chart of body weight of rats; **c** Statistical chart of 24 h urine output in rats; **d** Statistical chart of rat bladder weight; **e** Statistical chart of rat bladder capacity; **f** Statistical chart of average residual urine volume in rats; **g** Statistical chart of single urine output in rats; **h** Statistical chart of average urine output in rats; **i** Statistical chart of maximum pressure in the rat bladder; **j** HE staining of bladder tissue sections (× 100); **k** RT-qPCR was used to detect the relative expression level of miR-128 in bladder tissue. * indicates that compared with the NC group, P < 0.05, # indicates that compared with the PU group, P < 0.05. The above results are all measurement data, expressed as mean ± standard deviation. One-way ANOVA is used for comparison of data between multiple groups. Tukey’s post hoc test is performed, n = 8

The results of urodynamic testing under anesthesia showed that when STZ induced DM at 6 W and 12 W (Fig. 1e), compared with the NC group, the bladder volume of the rats in the PU group and the DM group increased significantly (P < 0.05) with the higher in the DM group (P < 0.05). In contrast to the NC group, the average residual urine of the PU group and the DM group rats was significantly increased (P < 0.05). Compared with the PU group, the residual urine volume of the DM group was significantly increased (P < 0.05), and it was further significantly increased at 12 W (P < 0.05) (Fig. 1f). At 6 W and 12 W, diabetes was induced by STZ (Fig. 1g), the single-time urine output of the rats in the PU group was more than that in the NC group (P < 0.05), and there was no significant difference compared with the single-time urine output of the DM group. The single-time urination volume at 6 W was significantly increased compared with the NC group (P < 0.05), and the difference was not significant at 12 W. The average urination rate results were shown in Fig. 1h. At 6 W, the average urination rate of rats in the DM and PU groups was not significantly different from that of the NC group. At 12 W, the average urination rate of the DM group was significantly lower than that of the NC group (P < 0.05). No significant difference was observed in the rate of urinary in the PU and NC group. At the same time, at 6 W and 12 W, compared with the NC group, the maximum bladder pressure in the DM group was significantly lower than that in the PU group, but no significant difference was observed in the PU group (Fig. 1i).

The HE staining results showed that in rats of the NC group and the PU group, the muscle bundles of the detrusor transverse and longitudinal cuts were neatly arranged, the muscle bundles were tightly structured, the gap was filled with connective tissue, the nerve bundles were more common, and the smooth muscle cells were arranged neatly with tight intercellular structure. In the DM group, the detrusor muscle bundles was disordered, the structure was loose, the muscle bundles was broken, the gap between muscle bundles was significantly widened, edema, lymphocyte infiltration, collagen fibers between muscle bundles were reduced, small blood vessels were congested, nerve The bundles were visible, muscle cells atrophied (Fig. 1j).

In addition, RT-qPCR was used to detect the expression of miR-128 in bladder tissues of rats in each group. The results showed that, under the same treatment time, miR-128 mRNA expression in bladder tissues of rats in the PU group and NC exhibited no significant difference, while the expression of miR-128 in bladder tissue of rats in the DM group was significantly higher than that of the NC group (P < 0.05), and was significantly higher at 12 W than at 6 W (P < 0.05) (Fig. 1k). The above results indicate that a rat diabetic bladder lesion model and a corresponding control model have been successfully constructed, and that miR-128 is highly expressed in the bladder tissue of a diabetic bladder lesion model rat, which may play a role in the occurrence of the lesion.

### Inhibition of miR-128 can improve the occurrence of diabetic bladder disease in rats

In order to study the effect of miR-128 expression on bladder lesions in DM rats, we selected a rat model injected with lentivirus. First, from the results of blood glucose and weight measurement, it was found that compared with the mimic NC group and the inhibitor NC group, the average blood glucose level of rats in the miR-128 mimic group was increased (P < 0.05), while that of rats in the 128 inhibitor group was reduced. There was no significant change in blood glucose levels between the mimic NC group and the inhibitor NC group (Fig. 2a). Compared with the weight of rats in the mimic NC group and inhibitor NC group, the weight of rats in the miR-128 inhibitor group was increased, and that in miR-128 mimic group was decreased compared with that of the mimic NC group (P < 0.05) (Fig. 2b).

**Fig. 2:** Inhibition of miR-128 improves the occurrence of diabetic bladder lesions in rats. **a** Statistical chart of blood glucose levels in rats; **b** Statistical chart of body weight of rats; **c** Statistical chart of 24 h urine output in rats; **d** Statistical chart of rat bladder capacity; **e** Statistical chart of average residual urine output in rats; **f** Statistical chart of single urine output of rats; **g** Statistical chart of average micturition rate of rats; **h** Statistical chart of maximum pressure in the bladder of rats; **i** Statistical chart of rat bladder weight).** J** Rat bladder tissue were observed by HE staining (× 100). * Indicates that compared with the mimic NC group P < 0.05, # indicates that compared with the inhibitor NC group P < 0.05. The above results are measured data, expressed as mean ± standard deviation. One-way ANOVA is used to compare data between multiple groups. Tukey’s post hoc inspection, n = 8

Urine was collected through a metabolic cage (Fig. 2c). Compared with the mimic NC group and inhibitor NC group, the daily urine output of rats in the miR-128 inhibitor group was significantly reduced, while increased in the miR-128 mimic group (P < 0.05). The bladder function of the mice in each group was subsequently examined by urodynamics, and the results showed that compared with the mimic NC group, t in the miR-128 mimic group, bladder volume (Fig. 2d), average residual urine volume (Fig. 2e), and single urination volume (Fig. 2f) all significantly increased (P < 0.05), but mean urination rate (Fig. 2g) and maximum bladder pressure (Fig. 2h) were decreased in the 12th week of STZ injection (P < 0.05), while it was opposite in miR-128 inhibitor group in comparison to the inhibitor NC group (P < 0.05).

After urodynamic examination, the bladder weight of each group of rats was excised and it was found (Fig. 2i) that compared with the mimic NC group and inhibitor NC group, the bladder weight of rats in the miR-128 inhibitor group was significantly reduced (P < 0.05), and that in rats in the miR-128 mimic group significantly increased (P < 0.05). The results of HE staining showed that compared with the mimic NC or inhibitor NC group, in the miR-128 mimic group, submucosal eosinophil infiltration was visible in the bladder wall, Severe mucous-like mucosa became smaller, swells, detrusor muscle cell morphology, size and disorder were arranged, smooth muscle tissue showed a large amount of collagen reduction and fiber dialogue, and interstitial fibrous tissue hyperplasia. In the miR-128 inhibitor group, detrusor muscle cells were arranged in an orderly manner, no significant degeneration of the myometrium was observed, and swelling was reduced (Fig. 2j). The above results indicate that overexpression of miR-128 can promote the occurrence of diabetic bladder disease in rats.

### miR-128 targets CB1 expression

In order to study the targeting relationship of miR-128 in bladder epithelial cells, first, we jointly predicted the downstream target genes of miR-128 through the bioinformation website microT, TargetScan, miRWalk and RNAInter, and took the intersection of the four predicted results to obtain 51 candidate genes (Fig. 3a). The STRING website was used to analyze the interactions between 51 candidate genes and the results was visualized using Cytoscape 3.5.1. We found that ITPKC and CNR1 (CB1) were at the core of the interaction network diagram (Fig. 3b). Through the analysis of TargetScan website, we found that miR-128 can target CB1 and predicted the binding site (Fig. 3c). Then, the prediction result of dual luciferase reporter gene assay (Fig. 3d) showed that compared with the mimic NC group, the luciferase activity of CB1 Wt 3′UTR was inhibited by miR-128 (P < 0.05), while CB1 Mut 3′UTR exhibited no change (P < 0.05). The results of RIP experiments showed that compared with IgG, both miR-128 and CB1 bound by Ago2 were significantly increased, indicating that miR-128 can specifically bind CB1′s 3′UTR region and down-regulates CB1 gene expression at post-transcriptional levels (Fig. 3e).

**Fig. 3:** miR-128 targets CB1 expression. **a** Venn diagram of bioinformation website microT, TargetScan, miRWalk and RNAInter predicting the intersection of downstream target genes of miR-128; **b** STRING website analyzes the interaction relationship network diagram of 51 candidate genes, circled in the figure Degree from large to small indicates the Degree of the gene, circle color from blue to orange indicates Degree from large to small, and the line in the middle of the circle indicates the co-expression relationship between genes; **c** Biology website predicts the binding position of miR-128 and CB1 Points; **d** Fluorescent activity detection results of miR-128 and CB1, * indicates comparison with the mimic NC group P < 0.05; **e** RIP experiments detect the binding of miR-128 and CB1 with Ago2, * indicates comparison with the anti-IgG group P < 0.05; **f** RT-qPCR detects the relative expression level of CB1 in bladder tissue, * indicates compared with NC group P < 0.05, # indicates compared with PU group P < 0.05; **g** miR-128 and CB1 correlation analysis; **h** RT-qPCR detection of each group Relative expression level of CB1 in rat bladder tissue; **i** Western blotting detection of CB1 protein expression level in rat bladder tissue in each group; **j** CB1 protein expression level statistical map. (**h**–**j**) * indicates that compared with the mimic NC group P < 0.05, # indicates that compared with the inhibitor NC group P < 0.05 The above results are measured data, expressed as mean ± standard deviation. Paired T test. One-way ANOVA was used to compare data between multiple groups. Tukey’s was used for post hoc tests

Then, we used RT-qPCR to detect the expression of CB1 in the bladder tissues of each group of rats, and the results (Fig. 3f) showed that compared with the NC group and the PU group, CB1 was poorly expressed in the bladder tissues of rats of the DM group. Moreover, correlation analysis showed that miR-128 was negatively correlated with CB1 expression in bladder tissues of DM rats (Fig. 3g). Subsequently, by interfering with the expression of miR-128, we used RT-qPCR and Western blotting to detect the mRNA and protein expression of CB1 in the bladder tissues of rats in each group (Fig. 3h–j). Compared with the mimic NC group, the mRNA and protein expression levels of CB1 in the miR-128 mimic group were significantly reduced (P < 0.05). Compared to the inhibitor NC group, the mRNA and protein levels of CB1 in the miR-128 inhibitor group were significantly increased (P < 0.05). In diabetic bladder disease tissues, miR-128 can target down-regulation of CB1 expression.

### miR-128 targets CB1 to regulate the occurrence of diabetic bladder disease

To study the role of CB1 expression in the development of diabetic bladder disease, we divided the DM rats into the following three groups for injection treatment: mimic NC + oe-NC group, miR-128 mimic + oe-NC group and miR-128 mimic + oe-CB1 group. qPCR was used to detect the expression of miR-128 in bladder tissues of rats in each group, qPCR and Western blotting were used to detect the expression of CB1 mRNA and protein in bladder tissues of rats in each group. Compared with the mimic NC + oe-NC group, in the bladder tissues of rats in the miR-128 mimic + oe-NC group, the expression of miR-128 significantly increased (P < 0.05) (Fig. 4a), and the mRNA and protein expression of CB1 significantly decreased (P < 0.05) (Fig. 4b, c). Compared with miR-128 mimic + oe-NC group, miR-128 mimic + oe-CB1 group had no significant change in miR-128 expression, and CB1 mRNA and protein expression increased significantly (P < 0.05) (Fig. 4b, c).

**Fig. 4:** Promoting effects of high expression of CB1 on miR-128 on diabetic bladder disease. **a** qPCR detects the expression level of miR-128 in bladder tissues of each group of rats; **b**, **c**. qPCR and Western blotting detection of the level of CB1 mRNA and protein in bladder tissues of each group of rats; **d** Statistics of blood glucose levels in rats; **e** Rat weight statistics; **f** Rat 24 h urine volume statistics; **g** Rat bladder volume statistics; **h** Rat average residual urine volume; **i** Rat single urine output statistics **j** Statistical chart of average micturition rate in rats; **k** Statistical chart of maximum pressure in the rat bladder; **l** Rat bladder weight and bladder tissue section HE staining (× 100). * Indicates that compared with the mimic NC + oe-NC group P < 0.05, # indicates that compared with the miR-128 mimic + oe-NC group, P < 0.05. The above results are all measurement data, expressed as mean ± standard deviation. Comparison of data between multiple groups using one-way ANOVA, Tukey’s post hoc test, n = 8

According to the results of blood glucose and weight measurement, it was found that compared with the mimic NC + oe-NC group, the average blood glucose level of rats in the miR-128 mimic + oe-NC group was significantly increased at the same experimental time (P < 0.05) (Fig. 4d), and the body weight was significantly reduced (P < 0.05) (Fig. 4b). In the miR-128 mimic + oe-CB1 group, the blood glucose level of the rats was significantly reduced (P < 0.05) (Fig. 4a), and the body weight was significantly increased (P < 0.05) (Fig. 4e). Urine was collected through a metabolic cage, and the results showed that compared with the mimic NC + oe-NC group, the daily urine output of rats in the miR-128 mimic + oe-NC group was significantly increased (P < 0.05). And in the miR-128 mimic + oe-CB1 group, the daily urine volume of rats was significantly reduced (P < 0.05) (Fig. 4f).

Subsequently, the bladder function of the mice in each group was examined by urodynamics. The results showed that, compared with the mimic NC + oe-NC group, in the miR-128 mimic + oe-NC group at 12 weeks of STZ injection, the mean maximum bladder volume, mean residual urine volume, and single voiding capacity all increased significantly (P < 0.05), and the maximum bladder pressure and mean micturition rate were significantly reduced (P < 0.05). Compared with the miR-128 mimic + oe-NC group, the mean maximum bladder volume (Fig. 4g), average residual urine volume (Fig. 4h), and single micturition volume (Fig. 4i) in rats of the 128 mimic + oe-CB1 group all significantly decreased (P < 0.05), and the maximum pressure in the bladder (Fig. 4j) and the mean micturition rate was significantly increased (P < 0.05) (Fig. 4k). After urodynamic examination, the bladder weight of each group of rats was excised and it was found that compared with the mimic NC + oe-NC group, the miR-128 mimic + oe-NC group had significantly increased bladder weight (P < 0.05). Compared with the miR-128 mimic + oe-NC group, the bladder weight of rats in miR-128 mimic + oe-CB1 group was significantly reduced (P < 0.05).

The results of HE staining showed that compared with the mimic NC + oe-NC group, in the miR-128 mimic + oe-NC group, the detrusor muscle bundles were disordered and loose, the muscle bundles were broken, and the gap between the muscle bundles was significantly widened, and urinary muscle cells atrophy, diverse morphology, lymphocyte infiltration, a large number of vacuolar degeneration, a small amount of eosinophilic degeneration, and increased interstitial and collagen components were observed. Compared with the miR-128 mimic + oe-NC group, in the miR-128 mimic + oe- CB1 group, the detrusor muscle bundles were arranged neatly, the structure was tight, the gap was filled with connective tissue, the muscle cells were vacuolated and the lymphocytes were infiltrated (Fig. 4l). The above results indicate that high expression of CB1 antagonizes the effect of miR-128 on the development of diabetic bladder disease.

### miR-128 regulates NF-KB/p-JNK axis through CB1 to affect the occurrence of diabetic bladder disease

In order to further study the regulatory mechanism of miR-128 on the occurrence of diabetic bladder disease through CB1, we found 414 genes related to diabetic bladder disease through the GeneCards database, analyzed the gene interaction using the STRING website, and found the gene NF-KB (NFKB1) can regulate p-JNK (MAPK8) to affect diabetic bladder disease (Fig. 5a). The co-expression relationship between CB1 and NF-KB in blood was obtained through the website Chipbase v2.0 (Fig. 5b), and the co-expression relationship between NF-KB and p-JNK (Fig. 5c). We know from the literature that CB1 can inhibit the activation of NF-KB [21], and NF-KB can promote the occurrence of diabetic bladder disease [22], and at the same time can promote the activation of JNK (p-JNK) [23] and activate JNK (p-JNK) can promote the occurrence of diabetic bladder disease by positively regulating apoptosis [24]. Therefore, we next explored that in the diabetic bladder, miR-128 regulates the NF-KB/p-JNK axis through CB1.

**Fig. 5:** miR-128 regulates NF-KB/p-JNK axis through CB1 to affect the occurrence of diabetic bladder disease. **a** STRING website analysis of gene interaction network diagram; **b**–**d** Western blotting detection of NF-KB and p-JNK and apoptosis in bladder tissue of three groups of NC, PU and DM rats Expression of related protein Bcl2, * indicates compared with NC group P < 0.05; **e** Western blotting detected NF-KB in rat bladder tissue of mimic NC group, miR-128 mimic group, inhibitor NC group and miR-128 inhibitor group, P-JNK and apoptosis-related protein Bcl2 expression, * indicates compared with mimic NC group P < 0.05, # indicates compared with inhibitor NC group P < 0.05; **f** Expression of NF-KB, p-JNK and apoptosis-related protein Bcl2 in bladder tissue of rats in each group by Western blotting, * indicates compared with the mimic NC + oe-NC group P < 0.05, # indicates compared with the miR-128 mimic + oe-NC group P < 0.05. **g** qPCR was used to detect the expression level of miR-128 in bladder tissue of rats in each group, * indicates compared with mimic NC + DMSO group P < 0.05; **h** qPCR detection of CB1 expression in bladder tissues of rats in each group, * indicates compared with mimic NC + DMSO group P < 0.05; **i** Western blotting detection of CB1, NF-KB, p-JNK and apoptosis-related protein Bcl2 in rat bladder tissue of each group Expression, * indicates compared with the mimic NC + DMSO group P < 0.05, # indicates compared with the miR-128 mimic + DMSO group P < 0.05; **j** statistical map of blood glucose levels in rats; **k** statistical map of body weights in rats; **l** 24 h urine volume statistics of rats; **m** bladder volume statistics of rats; **n** Statistics chart of average residual urine volume in rats; **o** Statistics chart of single urine output of rats; **p** Statistics chart of average urine output of rats; **r** Rat bladder weight statistics; **s** Bladder tissue section HE staining (× 100). Figure **j**–**r**, * indicates the comparison with mimic NC + DMSO group P < 0.05, # indicates the comparison with miR-128 mimic + DMSO group P < 0.05. The above results are all measurement data, expressed as mean ± standard deviation. One-way ANOVA and Tukey’s post hoc test was used to compare data between multiple groups

First, we detected the expression of NF-KB, p-JNK, and apoptosis-related protein Bcl2 in bladder tissue of NC, PU, and DM groups by Western blotting. The results showed that compared with the NC group, expressions of NF-KB p50, p-JNK and Bcl2 in the bladder tissues of the rats in the PU group were not significantly changed, but increased in the bladder tissues of rats in the DM group (P < 0.05) (Fig. 5d). Western blotting revealed that compared with the inhibitor NC group, the expression of NF-KB p50, p-JNK and Bcl2 in the bladder tissues of rats in miR-128 mimic group significantly increased, but that in the miR-128 inhibitor group were decreased (P < 0.05) (Fig. 5e). Moreover, compared with the miR-128 mimic + oe-NC group, the expression of NF-KB p50, p-JNK and Bcl2 were significantly decreased in the miR-128 mimic + oe-CB1 group (P < 0.05) (Fig. 5f). The above results indicate that miR-128 can regulate the expression of NF-KB and p-JNK through CB1 in the diabetic bladder and affect the level of apoptosis.

Further, after treated with miR-128 mimic, rats were simultaneously injected with NF-KB inhibitor PDTC, and Western blotting was used to detect NF-KB, p-JNK and apoptosis-related protein Bcl2 in bladder tissues of each group of rats expression. Rats were examined with urodynamics, and bladder tissue staining was performed. Compared with the mimic NC + DMSO group, in the bladder tissues rats in the miR-128 mimic + DMSO group, the expression of miR-128 increased significantly (P < 0.05) (Fig. 5g), mRNA and protein expression of CB1 was significantly reduced (P < 0.05) (Fig. 5h, i), and levels of NF-KB, p-JNK and Bcl2 were significantly increased (P < 0.05) (Fig. 5i), the mean blood glucose level was significantly increased (P < 0.05) (Fig. 5j), weight was significantly reduced (P < 0.05) (Fig. 5k), and the daily urine output was significantly increased (P < 0.05) (Fig. 5l), and the average maximum bladder volume (Fig. 5m), average residual urine volume (Fig. 5n), single urination volume (Fig. 5o) increased significantly (P < 0.05), mean micturition rate (Fig. 5p) and maximum bladder pressure (Fig. 5q) decreased significantly (Fig. 5m) (P < 0.05), the bladder weight increased significantly (P < 0.05) (Fig. 5r). Compared with the miR-128 + DMSO group, in the miR-128 mimic + PDTC group, the expression of miR-128 and CB1 were not significant changed in rat bladder, the expression of NF-KB, p-JNK and apoptosis-related protein Bcl2 were significantly reduced (P < 0.05) (Fig. 5i), and the body weight of rats was significantly increased (P < 0.05) (Fig. 5k), the average blood glucose level. Significantly decreased (P < 0.05) (Fig. 5j), daily urine output was significantly reduced (P < 0.05) (Fig. 5l), average maximum bladder volume (Fig. 5m), average residual urine volume (Fig. 5n), single urine output (Fig. 5o) were significantly decreased (P < 0.05), mean urination rate (Fig. 5p) and maximum bladder pressure (Fig. 5q) were significantly increased (P < 0.05), and bladder weight was significantly reduced (P < 0.05) (Fig. 5r).

The results of HE staining showed that compared with the mimic NC + DMSO group, the detrusor muscle bundles in the miR-128 mimic + DMSO group were disordered and loose, the muscle bundles were broken, the space between muscle bundles was significantly widened and edema, and the detrusor muscle cells atrophied, with diverse morphology, lymphocyte infiltration, and a large number of vacuolar degeneration observed. Compared with the miR-128 mimic + DMSO group, in the miR-128 mimic + PDTC group, detrusor muscle bundles were arranged more neatly, the structure was tight, and the gap was filled with connective tissue, with vascular degeneration of muscle cells and a small amount of lymphocyte infiltration found (Fig. 5s). The above results indicate that miR-128 regulates the NF-KB/p-JNK axis through CB1 and affects the occurrence of diabetic bladder disease.

## Discussion

Many miRNAs have been found to play important roles in DCP by regulating cytokines and then regulating tumor cell proliferation, metastasis, invasion and apoptosis. The role of miRNAs in cancer development has not been elucidated, and the role of miR-128a expression in diabetes is unclear, the corresponding regulatory mechanisms and downstream regulatory signals need further study. Even though the study of HIV-1 found that anti-miR-128 partially neutralized IFN-mediated HIV-1 blockade and elucidated the mechanism by which miR-128 impairs HIV-1 replication may provide new candidates for the development of therapeutic intervention [25]. And studies have shown that miR-128 levels are elevated in benign prostate epithelial cell lines compared to invasive prostate cancer cells. Knockdown of miR-128 can induce benign prostate epithelial cell infiltration, while overexpression of miR-128 attenuates infiltration of prostate cancer cells [26]. It has been reported that pro-neuron miR-128 is a candidate miRNA for glioma tumor suppressor. Reduced miR-128 expression is associated with aggressive human glioma subtypes. miR-128 has a tumor suppressive effect. miR-128 inhibits giNSC growth by enhancing neuronal differentiation. miR-128 inhibits growth and mediates differentiation by targeting oncogenic receptor tyrosine kinase (RTK) epithelial growth factor receptor and platelet-derived growth factor receptor alpha. [12] miR-128 is a glioma tumor suppressor that targets RTK signaling to inhibit giNSC self-renewal and enhance differentiation [27]. These results suggest that miR-128 plays a key role in DCP.

The miR-128 precursor can promote cell proliferation and inhibit apoptosis. Compared with the lnc-LAMC2-1: 1 rs2147578C allele, the G allele increases the risk of ovarian cancer by reducing the binding between lnc-LAMC2-1: 1 and miR-128-3p, thereby further reducing DCC and inhibition of apoptosis [28]. Myostatin (MSTN) inhibits excessive cardiac autophagy by blocking AMPK/mTOR and miR-128/PPARγ/NF-κB signaling pathways, at least partially significantly inhibiting pathological cardiac hypertrophy and dysfunction [29]. miR-128 can regulate the role and mechanism of glioma tumor angiogenesis through the miR-128/p70S6K1 axis, and miR-128 may become a potential therapeutic target for glioma in the future [13]. We predict that miR-128 targets the regulation of CB1 expression through bioinformatics, and through our findings, we found that miR-128 is highly expressed in the bladder tissue of diabetic bladder disease rats, and may play a role in the occurrence of lesions, And we found that by effectively inhibiting miR-128, we can improve the occurrence of diabetic bladder disease in rats. This is related to the abnormal expression of miRNAs (such as miR-128 and miR-21) in gliomas. In addition, there are reports in the literature that miR-128 is related to the proliferation of glioma cells, and that it reduces the expression of miR-10b [30], which can cause cell apoptosis. Existing studies have shown that miR-128 is highly expressed in central nervous cells but low in malignant gliomas. MiR-128 is a direct-acting target of P53 [31] and can interact with cyclins CDK6, BCL-2 and E2F3 form a complex that inhibits the translation of the target gene or degrades the miRNA of the target gene, induces the cell cycle to stagnate in the S phase, resulting in apoptosis and senescence [14]. These results suggest that we have a deeper understanding of miR-128. We adopt miR-128 inhibition to significantly improve the occurrence of diabetic bladder disease in rats and we have found for the first time that miR-128 can target the inhibition of CB1 expression. Previous studies have shown that CB1 can cause Inflammation, inflammation plays an important role in the development of diabetes [27]. Our high expression of CB1 can antagonize the promotion of miR-128 on the occurrence of diabetic bladder disease. qPCR and Western blotting were used to detect the expression levels of CB1 mRNA and protein in bladder tissue of rats in each group. Compared with the mimic NC + oe-NC group, miR-128 increased expression (Fig. 4a), CB1 mRNA and protein expression levels significantly decreased. CB1 mRNA and protein expression levels decreased significantly (Fig. 4b, c), compared with miR-128 mimic + oe-NC group, bladder tissue of rat was no significant change in miR-128 expression, and mRNA and protein expression levels of CB1 significantly increased (Fig. 4b, c). CB1 and our results show that miR-128 has significant regulatory role. Such results suggest that in the diabetic bladder, miR-128 may regulate the expression of signaling pathways NF-KB and p-JNK by regulating CB1. Previous studies have investigated the role of CB1 receptors in mediating 2-AG neuro protection. The findings suggest that 2-AG exerts its neuroprotective effect at least in part after CHI through the CB1 receptor-mediated mechanism, which involves inhibiting intracellular inflammatory signaling pathways [21]. Compared with previous studies, our research found that miR-128 regulates the NF-KB/p-JNK axis through CB1 to affect the occurrence of diabetic bladder disease.

## Conclusion

In summary, we report for the first time that miR-128 regulates the NF-KB/p-JNK axis through CB1 to affect the occurrence of diabetic bladder disease. We suggest further research on drugs with similar pharmacological characteristics to lay a theoretical foundation for an in-depth understanding of the pathogenesis of diabetic bladder disease and for finding new therapeutic targets.

## Data Availability

The authors confirm that the data supporting the findings of this study are available within the article.

## Abbreviations

DCP: Diabetic cystitis
DM: Diabetic Mellitus
NC: Normal control
STZ: Streptozotocin
PMSF: Phenylmethylsulfonyl fluoride
ANOVA: Analysis of variance
